# Prevalence of Postpartum Depression and Its Correlation With Breastfeeding in Makkah, Saudi Arabia: A Cross-Sectional Study

**DOI:** 10.7759/cureus.86037

**Published:** 2025-06-15

**Authors:** Rawan Zagzoog, Faisal Abdulrahman Alotaibi

**Affiliations:** 1 Public Health, Makkah Health Cluster, Ministry of Health Holdings, Makkah, SAU; 2 Public Health, Saudi Board of Preventive Medicine, Taif, SAU

**Keywords:** breastfeeding, edinburgh postnatal depression scale, postnatal period, postpartum depression, saudi arabia

## Abstract

Background

Postpartum depression (PPD) represents a significant public health concern with potential adverse effects on maternal well-being and infant development. Breastfeeding has been suggested to have a bidirectional relationship with PPD. This study aimed to assess the prevalence of PPD among Saudi women in Makkah and investigate its correlation with breastfeeding practices.

Methodology

A cross-sectional study was conducted among 378 postpartum mothers attending primary healthcare centres in Makkah, Saudi Arabia, between June and December 2024. The Edinburgh Postnatal Depression Scale (EPDS) was used to screen for PPD (score ≥12 indicating PPD). Data on sociodemographic characteristics, breastfeeding status, and duration were collected. Statistical analysis included descriptive statistics, chi-square tests, independent t-tests, analysis of variance, and logistic regression.

Results

The prevalence of PPD was 62.2% among the study population. The majority of participants (92.1%) were breastfeeding. No significant association was found between breastfeeding status and PPD prevalence (χ²(1) = 0.019, p = 0.891) or EPDS scores (t(376) = 0.243, p = 0.808). Breastfeeding duration showed no significant correlation with EPDS scores (r = -0.076, p = 0.138). In multivariate analysis, maternal age (odds ratio (OR) = 0.343, 95% confidence interval (CI) = 0.150-0.783 for 38-44 years) and cesarean delivery (OR = 1.752, 95% CI = 1.093-2.806) were significantly associated with PPD.

Conclusions

Despite previous literature suggesting a protective effect of breastfeeding against PPD, our findings indicated no significant association between breastfeeding practices and PPD in this Saudi population. The notably high prevalence of PPD (62.2%) compared to previous studies in Saudi Arabia warrants urgent attention from healthcare providers and policymakers. Maternal age and delivery mode emerged as significant factors, highlighting the need for targeted screening and interventions, particularly for younger mothers and those undergoing cesarean sections.

## Introduction

Postpartum depression (PPD) is a major mental health disorder that affects women during the postpartum period, typically within the first year after childbirth [1]. It is characterized by persistent feelings of sadness, anxiety, fatigue, and difficulties bonding with the newborn, significantly impacting maternal well-being and infant development [2]. The World Health Organization recognizes PPD as a significant public health concern affecting approximately 10-15% of women globally, though rates vary considerably across different populations and cultures [3].

Breastfeeding is universally recognized as the optimal method of infant feeding, providing numerous benefits for both mother and child. The World Health Organization, the European Commission Directorate for Public Health, and the American Academy of Pediatrics all recommend exclusive breastfeeding for the first six months of life [3-5]. The established benefits of breastfeeding include reduced risk of infections and diarrhea in infants, while mothers experience decreased risk of type 2 diabetes and uterine and ovarian cancers [6].

The relationship between breastfeeding and postpartum depression has been described as bidirectional. Research suggests that women with depression during pregnancy are less likely to plan to breastfeed [7], and those with PPD are less likely to initiate or continue breastfeeding [8]. Conversely, breastfeeding may protect against the development of PPD through various physiological and psychological mechanisms [9].

Physiologically, breastfeeding has been associated with improved maternal sleep patterns [10], attenuated stress responses [11], and anti-inflammatory effects that may protect against depression [12]. Studies have also reported that exclusive breastfeeding may help reduce depressive symptoms from childbirth to three months postpartum [9]. Furthermore, research has shown that breastfeeding may protect infants from the negative effects of maternal depression by preventing disengagement between mother and infant [13].

The prevalence of PPD varies widely across countries and sociodemographic groups. Studies from the United States have reported rates between 8.9% and 17% [14], while European studies show similar rates of approximately 13% [15]. In the Arab world, reported rates range from 10% in the United Arab Emirates [16], 16% in Lebanon [17], 17.8% in Saudi Arabia [18], and 22% in Northern Jordan [19].

Several factors have been associated with an increased risk of PPD, including maternal age, education level, income, employment status, mode of delivery, previous history of depression, and lack of social support [20]. However, there are inconsistencies in the literature regarding these associations, with some studies finding significant relationships while others do not [21].

In Saudi Arabia, studies on PPD have reported varying prevalence rates and associated factors. A study from the Eastern province found a prevalence of 17.8% [18], while another recent study from Al-Madinah reported a higher rate of 31.68% [22]. Research specifically examining the relationship between breastfeeding and PPD in Saudi Arabia is limited, creating a significant gap in understanding this relationship within the Saudi context.

Given the potential protective effects of breastfeeding against PPD and the considerable variation in findings across different populations, it is essential to investigate this relationship in the Saudi context. This study aims to assess the prevalence of PPD among Saudi women in Makkah and explore its correlation with breastfeeding practices. Understanding this relationship could inform targeted interventions to improve maternal mental health and promote optimal infant feeding practices in Saudi Arabia.

## Materials and methods

Study design and setting

This cross-sectional study was conducted in Makkah Al-Mokarramah, Saudi Arabia, from June 1, 2024, to December 30, 2024. Makkah contains approximately 85 primary healthcare centers (PHCCs) providing free health services to Saudi citizens. For this study, two sectors within Makkah were randomly selected, and from these sectors, two PHCCs were randomly chosen as the study sites.

Study population

The study targeted postpartum mothers attending obstetrics and gynecology (OBG) outpatient departments in the selected PHCCs for follow-up visits between four and eight weeks postpartum. Inclusion criteria were (1) women aged 18-45 years, (2) intention to breastfeed, and (3) having given birth to a full-term single infant. Exclusion criteria included (1) prenatal plans for exclusive formula feeding, (2) newborns admitted to neonatal intensive care for longer than 24 hours, (3) a history of depression, and (4) the presence of serious maternal medical conditions.

Sample size and sampling technique

The sample size was calculated using Epi-Info version 7 software. Based on a previous study reporting a 57.5% prevalence of PPD among pregnant women in Jeddah [23], with a confidence level of 95% and a precision of 5%, the minimum required sample size was determined to be 375 mothers.

A multi-stage stratified sampling technique was employed to ensure representativeness. In the first stage, Makkah was divided into nine districts based on administrative classifications, from which two districts were randomly selected. In the second stage, two PHCCs were randomly selected from these districts. In the third stage, the predetermined sample size was equally divided between the selected PHCCs, and mothers were randomly selected from each center.

Data collection tools

A comprehensive questionnaire consisting of two main components was used for data collection: Sociodemographic and clinical data: this section collected information on age, number of children, mode of delivery, previous miscarriages, education, employment status, monthly income, the presence of chronic diseases, intention to breastfeed, and the duration of exclusive breastfeeding. Edinburgh Postnatal Depression Scale (EPDS): this validated 10-item scale evaluates depressed mood experienced over the past week, with each item scored from 0 to 3 (minimum score 0, maximum 30). The Arabic version of the EPDS, previously validated in a sample of Emirati women [24], was used. Participants scoring ≤9 were categorized as having low risk, those scoring 10-11 as borderline, and those scoring ≥12 as having high risk for depression. Permission to use the Arabic version of the EPDS was obtained from the original developers or publishers before the commencement of the study.

Data collection procedure

Trained researchers approached potential participants in the waiting areas of the selected PHCCs. After explaining the study purpose, written informed consent was obtained from willing participants. The questionnaire was administered by the researcher, who was available to clarify any questions. Completed questionnaires were collected on the same day.

Ethical considerations

Ethical approval was obtained from the relevant ethics committee before data collection. All participants provided written informed consent after receiving a comprehensive explanation of the study goal, benefits, voluntary nature of participation, right to withdraw, and confidentiality measures. No personal identifiers were collected, and all data were used solely for research purposes.

Statistical analysis

Data were analyzed using SPSS version 28 (IBM Corp., Armonk, NY, USA). Normality of distribution was assessed using the Kolmogorov-Smirnov test. Descriptive statistics were presented as frequencies, percentages, means ± standard deviations, and medians with ranges. Reliability analysis was performed using Cronbach’s alpha. The chi-square test was used to examine the association between breastfeeding status and PPD prevalence. Independent t-tests were used to compare EPDS scores between breastfeeding and non-breastfeeding mothers, while one-way analysis of variance (ANOVA) was used to compare scores across different breastfeeding duration categories. Non-parametric alternatives (Mann-Whitney U test and Kruskal-Wallis test) were also performed for verification. Binary logistic regression was conducted to identify predictors of PPD, with the presence of PPD (EPDS score ≥12) as the dependent variable and sociodemographic factors, clinical characteristics, and breastfeeding practices as independent variables. Pearson’s and Spearman’s correlation analyses were performed to examine relationships between continuous variables. A p-value <0.05 was considered statistically significant for all analyses.

## Results

Sample characteristics

A total of 378 postpartum mothers participated in the study, with no missing data. The sociodemographic and clinical characteristics of the participants are presented in Table 1. The majority of participants (43.1%) were in the 28-37-year age group, followed by 38-44 years (31.7%), and 18-27 years (15.3%). All participants had children, with 63.8% having one to three children. Regarding delivery mode, 54.8% had vaginal deliveries, while 41.0% had cesarean deliveries. Nearly half (45.2%) of the participants reported previous miscarriages.

**Table 1:** Sociodemographic and clinical characteristics of participants (N = 378).

Characteristic	Category	Frequency	Percentage
Age (years)	18–27	58	15.3
	28–37	163	43.1
	38–44	120	31.7
	Not mentioned	37	9.8
Number of children	1–3	241	63.8
	4–6	120	31.7
	7–9	17	4.5
Mode of Delivery	Vaginal delivery	207	54.8
	Cesarean delivery	155	41.0
	Prefer not to answer	16	4.2
Previous miscarriage	Yes	171	45.2
	No	199	52.6
	Prefer not to answer	8	2.1
Education (years)	≤6	13	3.4
	6–12	80	21.2
	>12	285	75.4
Employment status	Employed	160	42.3
	Non-employed	205	54.2
	Not mentioned	13	3.4
Income (Saudi riyals)	<8,000	97	25.7
	8,000–15,000	87	23.0
	>15,000	53	14.0
	Not mentioned	141	37.3
Medical problems	Present	99	26.2
	Absent	271	71.7
	Not mentioned	8	2.1
Breastfeeding status	Yes	348	92.1
	No	30	7.9
Breastfeeding duration (months)	Did not breastfeed	30	7.9
	1	28	7.4
	<3	50	13.2
	3–6	65	17.2
	12	57	15.1
	13–18	78	20.6
	>18	70	18.5

Most participants (75.4%) had more than 12 years of education, and 54.2% were unemployed. Regarding income, 25.7% reported earning less than 8,000 SAR monthly, 23.0% earned between 8,000 and 15,000 SAR, and 14.0% earned more than 15,000 SAR. Medical problems were present in 26.2% of the participants.

All participants (100%) reported an intention to breastfeed. Among them, 348 (92.1%) were actively breastfeeding at the time of the study, while 30 (7.9%) were not. Regarding breastfeeding duration, 20.6% reported breastfeeding for 13-18 months, 18.5% for more than 18 months, 17.2% for 3-6 months, 15.1% for 12 months, 13.2% for less than 3 months, 7.4% for 1 month, and 7.9% had not breastfed.

Reliability and distribution of EPDS scores

The Arabic version of the EPDS demonstrated good internal consistency with a Cronbach’s alpha of 0.766. The mean EPDS score for the entire sample was 12.91 (SD = 5.30), with a median of 13.00 and scores ranging from 0 to 28. The 95% confidence interval (CI) for the mean was 12.37, 13.44. The distribution of EPDS scores showed a slight negative skewness (-0.08) and negative kurtosis (-0.228), indicating an approximately normal distribution. This was further confirmed by the Shapiro-Wilk test (p = 0.033) and Kolmogorov-Smirnov test (p = 0.069), which showed only a minor deviation from normality.

Prevalence of PPD

Based on the EPDS cutoff score of ≥12, the prevalence of PPD among the study participants was 235 (62.2%). Additionally, 44 (11.6%) scored in the borderline range (10-11), while 99 (26.2%) had scores below the threshold for depression (<10). The prevalence and categorization of PPD based on EPDS scores are presented in Table 2.

**Table 2:** Prevalence of postpartum depression based on EPDS scores (N = 378). EPDS: Edinburgh Postnatal Depression Scale

EPDS category	Frequency	Percentage
Negative (<10)	99	26.2
Borderline (10–11)	44	11.6
Positive (≥12)	235	62.2

Association between breastfeeding status and PPD

The chi-square analysis revealed no significant association between breastfeeding status and PPD prevalence (χ²(1) = 0.019, p = 0.891, Cramer’s V = 0.007). The PPD prevalence was nearly identical between non-breastfeeding (63.3%, 19/30) and breastfeeding mothers (62.1%, 216/348). Additionally, the independent t-test showed no significant difference in mean EPDS scores between non-breastfeeding (M = 13.13, SD = 5.55) and breastfeeding mothers (M = 12.89, SD = 5.29; t(376) = 0.243, p = 0.808, Cohen’s d = 0.046). Levene’s test confirmed homogeneity of variances (F = 0.126, p = 0.723). The non-parametric Mann-Whitney U test similarly showed no significant difference (U = 5054.0, Z = -0.289, p = 0.772), corroborating the t-test results.

Relationship between breastfeeding duration and EPDS scores

One-way ANOVA was conducted to examine differences in EPDS scores across breastfeeding duration categories. The results showed no significant differences (F(6, 371) = 0.687, p = 0.661, η² = 0.011). Levene’s test confirmed homogeneity of variances (F = 0.367, p = 0.899). The mean EPDS scores across breastfeeding duration categories are presented in Table 3.

**Table 3:** Mean EPDS scores by breastfeeding duration (N = 378). EPDS: Edinburgh Postnatal Depression Scale

Breastfeeding duration	N	Mean EPDS score	SD	Test statistic (F)
Did not breastfeed	30	13.13	5.55	F(6, 371) = 0.687
1 month	28	13.71	4.81	F(6, 371) = 0.687
<3 months	50	12.84	5.84	F(6, 371) = 0.687
3–6 months	65	13.78	5.45	F(6, 371) = 0.687
12 months	57	12.68	4.89	F(6, 371) = 0.687
13–18 months	78	12.68	5.13	F(6, 371) = 0.687
>18 months	70	12.16	5.40	F(6, 371) = 0.687

Post-hoc Tukey HSD tests revealed no significant pairwise differences between any of the breastfeeding duration groups. The largest mean difference was observed between the 3-6 months and >18 months groups (mean difference = 1.627, p = 0.564), while the smallest difference was between the 12 months and 13-18 months groups (mean difference = 0.001, p = 1.000).

Correlations between study variables

Pearson correlation analysis revealed a significant negative correlation between EPDS scores and maternal age (r = -0.224, p < 0.001, 95% CI = -0.316, -0.127), indicating that older mothers tended to have lower depression scores. This relationship was confirmed by non-parametric Spearman correlation (ρ = -0.200, p < 0.001). A weak positive correlation was found between breastfeeding duration and number of children (r = 0.128, p = 0.013, 95% CI = 0.027, 0.226), suggesting that mothers with more children tended to breastfeed slightly longer. As expected, a moderate positive correlation was observed between age and number of children (r = 0.470, p < 0.001, 95% CI = 0.389, 0.544). However, no significant correlation was found between EPDS scores and breastfeeding duration (r = -0.076, p = 0.138) or between EPDS scores and income (r = -0.029, p = 0.568) (Table 4).

**Table 4:** Correlations between study variables. EPDS: Edinburgh Postnatal Depression Scale

Variables	Correlation coefficient (r/ρ)	P-value	95% CI	Test used
EPDS score vs. maternal age	-0.224	<0.001	-0.316, -0.127	Pearson’s test
EPDS score vs. maternal age	-0.200	<0.001	N/A	Spearman’s test
Breastfeeding duration vs. number of children	0.128	0.013	0.027, 0.226	Pearson’s test
Age vs. number of children	0.470	<0.001	0.389, 0.544	Pearson’s test
EPDS score vs. breastfeeding duration	-0.076	0.138	N/A	Pearson’s test
EPDS score vs. income	-0.029	0.568	N/A	Pearson’s test

Predictors of PPD

Binary logistic regression analysis was performed to identify factors associated with PPD (EPDS score ≥12). The model included breastfeeding status, age, delivery mode, education level, employment status, and income as independent variables. The overall model was statistically significant (χ² = 29.811, df = 16, p = 0.019) and explained 10.3% of the variance in PPD status (Nagelkerke R² = 0.103). The Hosmer-Lemeshow test indicated good model fit (χ² = 3.545, p = 0.896).

Two variables emerged as significant predictors of PPD, namely, maternal age and delivery mode. Older mothers (38-44 years) had 65.7% lower odds of experiencing PPD compared to younger mothers (18-27 years) (odds ratio (OR) = 0.343, 95% CI = 0.150-0.783, p = 0.011). Cesarean delivery was associated with a 75.2% increase in the odds of PPD compared to vaginal delivery (OR = 1.752, 95% CI = 1.093-2.806, p = 0.020).

Breastfeeding status was not a significant predictor of PPD (OR = 1.228, 95% CI = 0.519-2.909, p = 0.640). Similarly, education level (p = 0.170), employment status (p = 0.299), and income (all categories p > 0.05) did not significantly predict PPD status. The results of the logistic regression analysis are presented in Table 5.

**Table 5:** Predictors of postpartum depression (N = 378). *: Statistically significant at p-values <0.05. OR: odds ratio; CI: confidence interval; Ref: reference category

Variable	Category	OR	95% CI	P-value
Maternal age (years)	18–27 (Ref)	1.00	-	0.008*
	28–37	0.561	0.265-1.186	0.130
	38–44	0.343	0.150-0.783	0.011*
Delivery mode	Vaginal (Ref)	1.00	-	0.038*
	Cesarean	1.752	1.093-2.806	0.020*
Breastfeeding status	No (Ref)	1.00	-	0.640
	Yes	1.228	0.519-2.909	0.640
Education level (years)	≤6 (Ref)	1.00	-	0.170
	6–12	1.458	0.399-5.325	0.568
	>12	0.871	0.253-2.997	0.827
Employment status	Employed (Ref)	1.00	-	0.299
	Non-employed	1.338	0.839-2.134	0.223
Income (SAR)	<8,000 (Ref)	1.00	-	0.632
	8,000–15,000	0.938	0.500-1.759	0.841
	>15,000	0.675	0.328-1.387	0.285

## Discussion

This cross-sectional study aimed to assess the prevalence of PPD among Saudi women in Makkah and explore its correlation with breastfeeding practices. Our findings revealed a strikingly high prevalence of PPD (62.2%) among the study population, substantially exceeding previously reported rates in Saudi Arabia and other regions. Contrary to some existing literature, we found no significant association between breastfeeding status or duration and PPD. Instead, maternal age and delivery mode emerged as significant predictors of PPD.

Prevalence of PPD

The 62.2% prevalence of PPD observed in our study is notably higher than previously reported rates in Saudi Arabia, which ranged from 17.8% in the Eastern province [18] to 31.68% in Al-Madinah [22]. It also substantially exceeds rates reported in other Arab countries, such as 10% in the United Arab Emirates [16], 16% in Lebanon [17], and 22% in Northern Jordan [19], as well as global estimates of 10-15% [3].

Several factors might contribute to this elevated prevalence. First, our study was conducted during 2025, a period that may still reflect long-term psychological impacts of the global COVID-19 pandemic, which has been associated with increased rates of perinatal mental health problems [25]. Second, methodological differences, including variations in screening tools, cut-off scores, and timing of assessment, may contribute to the disparities in reported prevalence rates [26]. Third, cultural factors specific to the Makkah region, such as family dynamics, postpartum practices, and societal expectations, might influence maternal mental health outcomes [27].

The high prevalence of PPD in our study underscores the urgent need for enhanced screening and mental health services for postpartum women in Makkah. It also highlights the importance of raising awareness about PPD among healthcare providers, families, and the broader community to reduce stigma and facilitate early intervention.

Breastfeeding and PPD

Contrary to our expectations and some previous research suggesting a protective effect of breastfeeding against PPD [8,9], our study found no significant association between breastfeeding status and PPD prevalence or EPDS scores. Moreover, there was no significant correlation between breastfeeding duration and depression scores, and breastfeeding status was not a significant predictor of PPD in the logistic regression analysis.

These findings align with some studies that reported no association between breastfeeding and PPD [28,29], suggesting that the relationship may be more complex than initially thought and potentially influenced by various contextual factors. Several explanations might account for our results.

First, the high rate of breastfeeding initiation (92.1%) in our sample reflects the strong cultural value placed on breastfeeding in Saudi society, which might be influenced by Islamic teachings encouraging breastfeeding for up to two years [30]. This cultural norm might result in women feeling pressured to breastfeed regardless of their psychological state, potentially masking any relationship between breastfeeding and depression.

Second, the bidirectional nature of the breastfeeding-depression relationship complicates interpretation. While breastfeeding might theoretically protect against depression through hormonal mechanisms [11], depression might also interfere with breastfeeding success and continuation [31]. These opposing effects might neutralize any observable association in cross-sectional studies such as ours.

Third, methodological factors, including the timing of assessment (four to eight weeks postpartum) and the cross-sectional design, limit our ability to capture the dynamic, temporal relationship between breastfeeding and PPD. A longitudinal approach would be more suitable for examining how changes in breastfeeding practices relate to changes in depressive symptoms over time.

Factors associated with PPD

Our logistic regression analysis identified two significant predictors of PPD, namely, maternal age and delivery mode. Older mothers (38-44 years) had significantly lower odds of experiencing PPD compared to younger mothers (18-27 years), consistent with several previous studies reporting higher vulnerability to PPD among younger mothers [21,32]. This age effect might be attributed to greater life experience, psychological maturity, and better coping strategies among older mothers [33].

Cesarean delivery was associated with a 75.2% increase in the odds of PPD compared to vaginal delivery, supporting previous findings linking cesarean sections to elevated PPD risk [34,35]. Several mechanisms might explain this association, including longer recovery periods, greater physical discomfort, complications from surgical procedures, and feelings of failure or disappointment when cesarean delivery was not planned [36]. Additionally, differential hormonal responses between vaginal and cesarean deliveries might influence maternal mood regulation [37].

Interestingly, other sociodemographic factors often associated with PPD, such as education level, employment status, and income, were not significant predictors in our study. This divergence from some previous findings might reflect the particular social context of Makkah, where cultural factors and social support systems might moderate the influence of these socioeconomic variables.

Strengths and limitations

This study has several strengths, including a large, representative sample from randomly selected primary healthcare centres, the use of a validated Arabic version of the EPDS, a comprehensive assessment of breastfeeding practices, and robust statistical analyses including both parametric and non-parametric approaches.

However, several limitations should be considered when interpreting our findings. First, the cross-sectional design precludes causal inferences regarding the relationship between breastfeeding and PPD. Second, the use of self-reported measures introduces the possibility of recall bias and social desirability bias, particularly given the cultural value placed on breastfeeding in Saudi society. Third, the timing of assessment (four to eight weeks postpartum) captures only one point in the dynamic postpartum period, potentially missing earlier onset of symptoms or changes in breastfeeding practices over time. Fourth, while the EPDS is a screening tool with good sensitivity and specificity, clinical diagnoses of PPD would require structured clinical interviews. Finally, our sample excluded women with a history of depression, potentially limiting the generalizability of our findings to the broader postpartum population.

Implications for practice and research

Our findings have several important implications for clinical practice, public health initiatives, and future research. For clinical practice, the alarmingly high prevalence of PPD (62.2%) highlights the critical need for routine screening of all postpartum women, preferably using validated tools such as the EPDS, during regular postpartum visits. Particular attention should be paid to younger mothers and those who have undergone cesarean deliveries, as these groups appear more vulnerable to PPD. Additionally, healthcare providers should be trained to recognize symptoms of PPD and be knowledgeable about appropriate referral pathways for further assessment and management.

From a public health perspective, there is an urgent need for enhanced mental health services specifically targeting postpartum women in Makkah. This might include specialized postpartum mental health clinics, telepsychiatry services for those unable to access in-person care, and community-based support groups. Public awareness campaigns about PPD, highlighting its prevalence, symptoms, and available resources, could help reduce stigma and encourage women to seek help.

For future research, longitudinal studies starting from pregnancy through the extended postpartum period would better capture the temporal relationship between breastfeeding and PPD. Qualitative research exploring women’s experiences of breastfeeding and postpartum mental health within the Saudi cultural context would provide valuable insights into the complex interplay of biological, psychological, and sociocultural factors. Additionally, intervention studies testing the effectiveness of various approaches to preventing and treating PPD in this population would be particularly valuable.

## Conclusions

This cross-sectional study found a strikingly high prevalence of PPD (62.2%) among women in Makkah, Saudi Arabia. Contrary to some previous literature, no significant association was observed between breastfeeding practices and PPD. Instead, maternal age and delivery mode emerged as significant predictors, with younger mothers and those who underwent cesarean deliveries at higher risk for PPD. These findings underscore the urgent need for enhanced screening, intervention, and support services for postpartum women in Makkah, with particular attention to vulnerable groups. While our study did not confirm a protective effect of breastfeeding against PPD, it highlights the complex, multifactorial nature of PPD and the importance of comprehensive approaches to maternal mental health that address biological, psychological, and sociocultural factors. Future longitudinal research is needed to better understand the temporal dynamics between breastfeeding and PPD in the Saudi context, as well as to develop and evaluate culturally appropriate interventions to support maternal mental health during this critical period.

## Figures and Tables

**Figure 1:** IRB letter
